The article "Aromaticity indices, electronic structural properties, and fuzzy atomic space investigations of naphthalene and its aza-derivatives" was retracted in 2026. Reasons: unreliable results or conclusions; concerns about the citations.

# Aromaticity indices, electronic structural properties, and fuzzy atomic space investigations of naphthalene and its aza-derivatives

**DOI:** 10.1016/j.heliyon.2021.e06138

**Published:** 2021-02-01

**Authors:** Moses M. Edim, Obieze C. Enudi, Bassey B. Asuquo, Hitler Louis, Emmanuel A. Bisong, John A. Agwupuye, Apebende G. Chioma, Joseph O. Odey, Innocent Joseph, Francisca I. Bassey

**Affiliations:** a Department of Chemistry, Faculty of Physical Sciences, Cross River University of Technology, Calabar, Nigeria; b Computational Quantum Chemistry Research Group, University of Calabar, Calabar, Nigeria; c Department of Pure and Applied Chemistry, Faculty of Physical Sciences, University of Calabar, Calabar, Nigeria; d Nanoscience, National Centre for Nanoscience and Technology, University of Chinese Academy of Sciences, Beijing, China

**Keywords:** Diazanaphthalenes, CDFT, Aromaticity, NBO, Structural

## Abstract

The aromaticity and CDFT properties of naphthalene and its aza-derivatives were theoretically investigated using density functional theory (DFT) electronic structure method. The reactivity and chemistry of Azanaphthalene (1-AN), 1, 2-diazanaphthalene (1, 2-DAN), 1, 3-diazanaphthalene (1, 3-DAN), 1, 4-diazanaphthalene (1,4-DAN), 1, 5-diazanaphthalene (1, 5-DAN), 1, 6-diazanaphthalene (1, 6-DAN), 1, 7-diazanaphthalene (1,7-DAN) and 1, 8-diazanaphthalene (1, 8-DAN) were thoroughly explored and predicted focusing more on the fuzzy atomic space analysis, quantum chemical descriptors (CDFT), natural bond orbital (NBO), and structural electronic properties. The CDFT is focused on predicting the condensed Fukui function and dual descriptors along with condensed local electrophilicity and nucleophilicity investigation. From the aromaticity computational study, 1,7-DAN gave PDI, FLU, FLU-π, PLR, HOMA, BIRD and LOLIPOP values of approximately one (1) was found to be the most aromatic in the group, and strongest π-stacking ability. The aromaticity follows the trend: 1, 7-DAN > 1, 8-DAN > 1, 5-DAN > 1, 6-DAN > 1, 4-DAN > 1, 2-DAN > 1-AN > naphthalene. The second order perturbation energy NBO analysis revealed that the 3 highest stabilization energies in the molecules are C_6_–N_a_ to C_3_–C_4_$(\pi^{*}-\pi^{*}$ 236.90 kcal/mol) of 1, 6-DAN, C_3_–C_4_ to C_1_–C_2_ ($\pi^{*}-\pi^{*}$236.37 kcal/mol) of 1-AN and C_7_–N_10_ to C_2_–C_4_ ($\pi^{*}-\pi^{*}$235 kcal/mol) of 1, 3-DAN.

## 1 Introduction

We encounter aromatics in our daily lives. The chemistry of our body would be distorted in the absence of aromatic molecules in our system, also, we would be lacking many materials needs. Many industrial raw materials are aromatics based, ranging from polymer, medicine and various other industries [1]. About 35 million tons of aromatic compounds are manufactured in the world every year to produce essential chemicals and polymers, such as polyester, nylon, vinyl polymers (e.g. styrene) etc. They also play essential biochemical roles in living systems [1, 2]. Naphthalene structurally consists of a fused pair of benzene rings sharing adjacent carbon atoms. Naphthalene, a component of petroleum has been applied in vertinary medicine, dusting powder and as an insecticide [3]. Aza derivatives of naphthalene are formed on the substitution of a carbon atom with nitrogen. The derivatized aza compounds are either mono-, di-, tri-etc. depending on the number of carbon atoms replaced by nitrogen [4]. The position(s) and number of nitrogen atom(s) in the ring confers chemical properties on the basic structure. Diazanaphthalenes are a broad class of N-heteroaromatic compounds with several technological and biological applications. They consist of a naphthalene double ring in which two of the carbon atoms have been replaced with Nitrogen atom. Positional isomers of diazanaphthalenes exists. The isomers differ by the locations of the nitrogen. The isomers are divided into two subgroups: benzodiazines and naphthyridines [5, 6]. The benzodiazines have both nitrogen atoms in one ring. They include; cinnoline, quinazoline, quinoxaline and phthalazine. While, the naphthyridines, which have one nitrogen atom per ring include 1,7-naphthyridine, 2,7-naphthyridine, 1,6-naphthyridine, 1,5-naphthyridine, 1,8-naphthyridine and 2,6-naphthyridine [5, 6, 7]. Diazanphthalenes have several uses and applications. For example, 1,8-naphthyridine derivatives have Medicinal properties such as anti-HIV, anti-cancer, anti-inflammatory, anti-malarial, anti-bacterial, anti-protozoans, anti-mycobacterial and anti-platelet [7]. Some of their applications of are attributed to their ability to form association dimers through non-covalent interactions [8, 9, 10].

The article "Aromaticity indices, electronic structural properties, and fuzzy atomic space investigations of naphthalene and its aza-derivatives" was retracted in 2026. Reasons: unreliable results or conclusions; concerns about the citations.

Modern computational chemistry is focused on obtaining exact data. However, obtaining exact data is still not achievable for majority of molecules. For most computational chemist, only approximate theoretical levels are accessible. On the other hand, there are several organic physical chemistry descriptors, such as aromaticity, solvents, substituents. Reactivity indices, etc., that can be used for modelling the properties of interest [11].

The Density-Functional Theory (DFT) is a computational quantum mechanical modelling method used to investigate the electronic structure of nuclear structure in atoms or molecules [12]. DFT computational codes are used in practice to investigate the structural, magnetic and electronic properties of molecules, materials and defects. In DFT, the functional is the electron density which is a function of space and time [13, 14]. The electron density is used in DFT as the fundamental property. The usefulness of electron density was further revealed by Hohenburg and Kohn. The Hohenburg-Khon theorem asserts that the density of any system determines all ground state properties of the system [15]. This implies that the total ground state energy of a many-electron system is a functional of the density [13]. Generally, DFT is applied in the interpretation and prediction of complex system behavior at an atomic scale [13, 15, 16, 17, 18].

Parr developed the conceptual DFT, a DFT sub-field, in the early 1980s [19]. In CDFT, one tries to extract important concepts and principles from the electron density of a molecule, such that their chemistry will be understood or predicted [19, 20]. Very relevant indices are derived using the conceptual DFT to study organic molecules, which the reactivity could be explained. The derivable parameters of electron density which are special tools in the determination of molecular reactivity are; chemical potential μ, electronegativity χ (opposite of μ), chemical hardness Ƞ and softness *S*, Fukui function f, etc. [21].

Aromaticity of organic compounds is one of the most important characteristics related to the specific chemical reactivity structure [22]. As a measure of aromaticity, many parameters based structural changes or electron densities can be used [23]. The purpose of this study is to provide information about the aromaticity of the polycyclic system of naphthalene and its aza-derivatives based on the structure. Naphtahlene is a dicyclic aromatic hydrocarbon, with formula C_10_H_8_. Aza derivatives of naphthalene are formed on the substitution of carbon atoms with nitrogen. It is particularly interesting to establish whether the azanaphthalenes can be more aromatic. The difference between some properties of naphthalene molecule is sensitive to the introduction of nitrogen atoms.

## 2 Computational details

All DFT quantum chemistry calculations were performed using the Gaussian 09 software [24], and the Gauss view 6.0 interface. All the ground state compounds were optimized using the DFT/B3LYP methods and the 6–311++G (d, p) basic set [25]. The natural bond orbital analysis was carried using Gaussian 09, and results analyzed using UCA Fukui software [26]. The electronic structure analysis of the conceptual DFT descriptors, Laplacian bond order, atomic charge, and aromaticity indices were performed using the Multiwfn 3.7 (dev) code [27], which can be freely obtained at the official website (http://sobereva.com/multiwfn). The ESP, DOS, isosurface, and the scanning tunneling microscope (STM) images were plotted for all compounds using the Visual Molecular Dynamics (VMD) software [28] based on the files exported by Multiwfn. In this study, the various compounds are coded thus; 1-AN = azanaphthalene, 1, 2-DAN = 1, 2-diazanaphthalene, 1, 3-DAN = 1, 3-diazanaphthalene, 1,4-DAN = 1, 4-diazanaphthalene, 1, 5-DAN = 1, 5-diazanaphthalene, 1, 6-DAN = 1, 6-diazanaphthalene, 1,7-DAN = 1, 7-diazanaphthalene and 1, 8-DAN = 1, 8-diazanaphthalene (see Figure 1).

The article "Aromaticity indices, electronic structural properties, and fuzzy atomic space investigations of naphthalene and its aza-derivatives" was retracted in 2026. Reasons: unreliable results or conclusions; concerns about the citations.

**Figure 1:** The Geometric Diagrams of Naphthalene, 1-AN, 1,2-DAN, 1,3-DAN, 1,4-DAN, 1,5-DAN, 1,6-DAN, 1,7-DAN AND 1,8-DAN showing their respective auto-assigned atom number by Gaussian 09 software.

## 3 Results and discussion

### 3.1 Conceptual density functional theory (CDFT)

This study investigates the effect of fused nitrogen atoms in the stability, aromaticity and reactivity indices of naphthalene, also, the reactive sites and their nature is determined using CDFT parameters. Here, the interest is the magnitude and trends in property values as we move from Naphthalene to the mono-substituted azanaphthalene, and also as amongst the diazanaphthalenes (1, 2-DAN, 1, 3-DAN, 1, 4-DAN, 1, 5-DAN, 1, 6-DAN, 1, 7-DAN AND 1, 8-DAN).

#### 3.1.1 Total energy (TE)

The energy of the optimized structures of the various species was calculated. as can be seen in Table 1, naphthalene and 1-AN possesses the highest total energy of -10,499.36 Kcal/mol at neutral states. A significant difference in total energy is visible between 1-AN and 1,2-DAN (i.e. 871.83 Kcal/mol), this could be an introduction of extra stability by the introduction of a second nitrogen atom into the ring structure. The lone pairs on the nitrogen atoms increase the electron density, which improves the resonance around the rings of the azanaphthalene and diazanaphthalene [29], hence gives a more stable molecule. A gradual decrease in total energy was observed for all diazanaphthalene compounds as the second nitrogen atom is moved around the ring to give 1,3-DAN, 1,4-DAN, 1,5-DAN, 1,6-DAN, 1,7-DAN and 1, 8-DAN (with the least TE observed for 1, 8-DAN: -11,375.00 Kcal/mol). This implies that 1,3-DAN, 1,7-DAN and 1, 8-DAN (with TE = -11, 379.88, -11,374.12 and -11,375.00 Kcal/mol, respectively) are more stable compounds at neutral state by virtue of their relative total energy values. Calculation were carried out for N+1 and N-1 states of the different species. From N+1 and N-1 values in Table 1, a trend of increasing stability is observed from normal naphthalene, 1-AN, 1,2-DAN to 1, 8-DAN. 1, 8-DAN also exhibited the lowest total energy at +1 and -1 states, making it more stable than other counterparts in ionic state. Aromaticity is generally manifested through high stability, low reactivity and low magnetic susceptibility [30]. From TE values in Table 1, Normal naphthalene and 1-AN show low aromaticity when compared to the diazanaphthalene counterparts, aromaticity thus has the following trend; naphthalene < 1-AN < 1,2-DAN< 1,3-DAN < 1,4-DAN < 1,5-DAN < 1,6-DAN < 1,7-DAN < 1, 8-DAN.

The article "Aromaticity indices, electronic structural properties, and fuzzy atomic space investigations of naphthalene and its aza-derivatives" was retracted in 2026. Reasons: unreliable results or conclusions; concerns about the citations.

**Table 1:** CDFT results showing the values of different property determined parameters for Naphthalene, 1-AN, 1,2-DAN, 1,3-DAN, 1,4-DAN, 1,5-DAN, 1,6-DAN, 1,7-DAN AND 1,8-DAN.

S/N	Property	Naphthalene	1-AN	1,2-DAN	1,3-DAN	1,4-DAN	1,5-DAN	1,6-DAN	1,7-DAN	1,8-DAN
1	Total Energy (N) (Kcal/mol)	-10,499	-10,499	-11,371	-11,380	-11,372	-11,372	-11,372	-11,374	-11,375
2	Total Energy (N+1)	-10,498	-10,498	-11,371	-11,371	-11,372	-11,373	-11,374	-11,374	-11,372
3	Total Energy (N-1)	-10,491	-10,491	-11,363	-11,363	-11,363	-11,364	-11,365	-11,368	-11,363
4	HOMO Energy (eV)	-6.15	-6.65	-6.53	-7.09	-7.05	-7.03	-7.08	-7.06	-7.08
5	LUMO Energy (eV)	-1.40	-1.82	-2.38	-2.22	-2.35	-2.20	-2.22	-2.24	-2.20
6	Energy Gap (eV)	4.75	4.23	4.83	4.87	4.70	4.83	4.87	4.83	4.90
7	Vertical IP (eV)	8.01	8.01	8.12	8.49	8.63	8.49	8.78	8.78	8.53
8	2nd Vertical IP (eV)	13.58	13.58	14.67	14.27	14.66	15.03	14.92	14.80	15.06
9	Electron Affinity (eV)	-1.19	-1.19	-0.36	-0.81	-0.28	-0.48	-0.46	-0.46	-0.46
10	Mulliken Electronegativity	3.41	3.41	3.88	3.84	4.17	4.01	4.16	4.16	4.03
11	Chemical Potential	-3.41	-3.41	-3.88	-3.84	-4.17	-4.01	-4.16	-4.16	-4.03
12	Hardness	9.19	9.19	8.47	9.30	8.91	8.97	9.24	9.24	8.99
13	Softness	0.11	0.63	0.01	0.01	0.01	0.01	0.11	0.11	0.01
14	Electrophilicity index	0.64	0.63	0.89	0.79	0.98	0.90	0.94	0.94	0.91
15	Nucleophilicity index	3.00	3.00	3.25	2.58	2.66	2.65	2.38	2.39	2.60
16	Cubic Electrophilicity index	0.83	0.83	1.00	0.99	1.15	1.04	1.12	0.41	1.05

#### 3.1.2 HOMO-LUMO/energy gap

Highest occupied molecular orbital and lowest unoccupied molecular orbital energy gap is one of the descriptors for reactivity [31]. The Energy gap is solely dependent on the values of HOMO and LUMO of the compound in context.

(1) Energy Gap (Δ*E*) = *E*_LUMO_ - *E*_*HO*MO_

Where; *E*_HOMO_ and *E*_LUMO_ are the energies of the HOMO and LUMO, respectively. Energy is usually reported in eV or Kcal/mol [4]. The HOMO energy is employed in the determination of ionization potential (IP), while the LUMO energy is used in the determination of many reactivity indices because it is related to several parameters, e.g. electron affinity (EA) [36]. Molecules with high band gap requires great energy for electron delocalization, so regarded to be less reactive [32]. 1-AN exhibited the least energy gap (4.229124 eV) as can be deduced from the HOMO and LUMO values in Figure 2. A high energy gap of 4.87 eV for 1,3-DAN and 1,6-DAN, depicts stability. Furthermore, 1, 8-DAN exhibits relatively the highest HOMO-LUMO energy gap value (4.90 eV), which explains its predicted stability with respect to energy configuration [33].

The article "Aromaticity indices, electronic structural properties, and fuzzy atomic space investigations of naphthalene and its aza-derivatives" was retracted in 2026. Reasons: unreliable results or conclusions; concerns about the citations.

**Figure 2:** The isosurface of the HOMO (3A) and LUMO (3A) for Naphthalene, 1-AN, 1,2-DAN, 1,3-DAN, 1,4-DAN, 1,5-DAN, 1,6-DAN, 1,7-DAN and 1,8-DAN showing their respective Energy.

The orbital indices gotten from Multiwfn [28] for HOMO and LUMO for all the compounds analyzed are 34 and 35 respectively. From the isosurface diagrams of the HOMO of the various compounds in Figure 2 similarities can be ascertained between naphthalene and 1-AN, where the HOMO orbital is evenly distributed around the ring. 1,2-DAN have its HOMO concentrated around the N–N bond. It is obvious from the HOMO diagrams of 1,7-DAN and 1, 8-DAN that their HOMO is concentrated on the nitrogen atoms, which are the reactive sites of the diazanaphthalenes. Rationally, it can be predicted from the visualized HOMO lobes, that the nitrogen sites are liable to accept point charges during electron delocalization. The LUMO of naphthalene, 1-AN, 1,2-DAN, 1,3-DAN, 1,4-DAN, 1,5-DAN, 1,6-DAN, 1,7-DAN and 1, 8-DAN are evenly distributed around their respective molecules.

#### 3.1.3 Ionization potentials (IP)

Vertical Ionization Potential (VIP) which is the amount of energy required for a species in gaseous phase to lose an electron. It can be theoretically calculated thus;

(2) VIP = E(N-1) – E(N)

Where; E(N-1) and E(N) are the electronic energies for a species at its charged (N-1) and neutral (N) states, respectively.

The vertical ionization potentials for naphthalene, 1-AN, 1, 2-DAN, 1, 3-DAN, 1, 4-DAN, 1, 5-DAN, 1, 6-DAN, 1, 7-DAN and 1, 8-DAN were calculated for the respective optimized structures using the Multiwfn software [27] and the results are reported in Table 1. It can be observed that Vertical IP increased from naphthalene to 1, 4-DAN, after which there is an irregular trend from 1, 2-DAN to 1, 8-DAN. 1, 6-DAN and I, 7-DAN gave the relatively highest IP values of 8.78 eV. But the distribution of Ionization potential is relatively slim (from the least 8.01 eV (form naphthalene and 1-AN) to the highest 8.78 (for 1, 6-DAN and 1, 7-DAN)). Though, 1, 6-DAN and 1, 7-DAN having the highest IP are more stable.

#### 3.1.4 Chemical hardness (Ƞ) and softness (S)

Chemical hardness is perceived as a molecule's resistance to exchange electron density with the immediate surrounding [34]. This is the reciprocal of chemical softness [40]. Both Ƞ and *S* were analyzed for all tested compounds employing the Multiwfn software [28], which invoked the regular expressions;

(3) *η* = VIP – VEA

Where; VIP is the Vertical Ionization Potential, VEA is the Vertical Electron Affinity.

The article "Aromaticity indices, electronic structural properties, and fuzzy atomic space investigations of naphthalene and its aza-derivatives" was retracted in 2026. Reasons: unreliable results or conclusions; concerns about the citations.

VIP is expressed in Eq. (2), while VEA can be calculated theoretically using the expression;

(4) VEA = *E*(N) – *E*(N = 1)

*S* is the reciprocal of η. The chemical hardness values of all species in Table 1, are closely dispersed. A chemical hardness value of 9.3005 shown by 1,3-DAN is the highest for the group, which implies that it is highly reluctant to exchange electron density with the environment. Both normal naphthalene and 1-AN showed same hardness value of 9.1924, hence the introduction of the first nitrogen atom didn't affect the hardness of naphthalene.

#### 3.1.5 Mulliken electronegativity (χ) and chemical potential (μ)

Electronegativity is the measure of the bonding electron withdrawing tendency of an atom or molecule [34]. It is the opposite of chemical potential.

(5) $$\chi =\left(\frac{VIP+VEA}{2}\right)$$

Chemical potential, which is the opposite of Mulliken electronegativity is derived by multiplying Eq. (5). by the negative sign (-) to yield;

(6) $$\mu =-\left(\frac{VIP+VEA}{2}\right)$$

As reported in Table 2, naphthalene and 1-AN show similarities in several properties, they also share same electronegativity value of 3.41. An appreciation in electronegativity is noticed for 1,2-DAN and 1,3-DAN (3.8791 and 3.8363 respectively). A significant increment is notable for 1,4-DAN (4.1715), which is the highest in the group, making 1,4-DAN the most electronegative of this group of compounds.

**Table 2:** Condensed Local Electrophilicity and Nucleophilicity (e∗eV) Indices for the various C and N atoms in Naphthalene, 1-AN, 1,2-DAN, 1,3-DAN, 1,4-DAN, 1,5-DAN, 1,6-DAN, 1,7-DAN AND 1,8-DAN.

		**C1**	**C2**	**C3**	**C4**	**C5**	**C6**	**C7**	**C8**	**C9**	**C10**
Electrophilicity	Naphthalene	0.05	0.05	0.01	0.05	0.01	0.05	0.05	0.05	0.05	0.05
Nucleophilicity		0.27	0.23	0.05	0.23	0.05	0.27	0.27	0.23	0.23	0.27
		**C1**	**C2**	**C3**	**C4**	**C5**	**C6**	**C7**	**C8**	**C9**	**N17**
Electrophilicity	1-AN	0.06	0.06	0.02	0.02	0.06	0.06	0.08	0.06	0.08	0.08
Nucleophilicity		0.32	0.27	0.05	0.06	0.18	0.03	0.14	0.23	0.18	0.16
		**C1**	**C2**	**C3**	**C4**	**C5**	**C6**	**C7**	**C8**	**N9**	**N10**
Electrophilicity	1,2-DAN	0.07	0.07	0.02	0.07	0.02	0.07	0.10	0.10	0.11	0.11
Nucleophilicity		0.12	0.26	0.26	0.26	0.26	0.12	0.25	0.25	0.13	0.13
		**C1**	**C2**	**C3**	**C4**	**C5**	**C6**	**C7**	**C8**	**N9**	**N10**
Electrophilicity	1,3-DAN	0.06	0.06	0.02	0.07	0.02	0.06	0.06	0.09	0.11	0.11
Nucleophilicity		0.08	0.17	0.18	0.18	0.13	0.11	0.25	0.23	0.61	0.63
		**C1**	**C2**	**C3**	**C4**	**C5**	**C6**	**C7**	**C8**	**N9**	**N10**
Electrophilicity	1,4-DAN	0.07	0.07	0.02	0.07	0.02	0.07	0.10	0.10	0.11	0.11
Nucleophilicity		0.12	0.26	0.26	0.26	0.26	0.12	0.25	0.25	0.13	0.13
		**C1**	**C2**	**C3**	**C4**	**C5**	**C6**	**C7**	**C8**	**N9**	**N10**
Electrophilicity	1,5-DAN	0.08	0.06	0.02	0.86	0.19	0.09	0.06	0.08	0.08	0.08
Nucleophilicity		0.12	0.15	0.10	0.20	0.10	0.20	0.15	0.12	0.42	0.43
		**C1**	**C2**	**C3**	**C4**	**C5**	**C6**	**C7**	**C8**	**N9**	**N10**
Electrophilicity	1,6-DAN	0.07	0.06	0.02	0.02	0.09	0.10	0.06	0.09	0.09	0.09
Nucleophilicity		0.11	0.13	0.09	0.09	0.17	0.17	0.13	0.11	0.33	0.43
		**C1**	**C2**	**C3**	**C4**	**C5**	**C6**	**C7**	**C8**	**N9**	**N10**
Electrophilicity	1,7-DAN	0.10	0.02	0.06	0.02	0.07	0.09	0.08	0.09	0.09	0.08
Nucleophilicity		0.16	0.09	0.13	0.09	0.13	0.18	0.13	0.11	0.32	0.44
		**C1**	**C2**	**C3**	**C4**	**C5**	**C6**	**C7**	**C8**	**N9**	**N10**
Electrophilicity	1,8-DAN	0.09	0.02	0.02	0.07	0.08	0.09	0.07	0.08	0.08	0.08
Nucleophilicity		0.19	0.10	0.10	0.14	0.13	0.19	0.14	0.13	0.39	0.39

The article "Aromaticity indices, electronic structural properties, and fuzzy atomic space investigations of naphthalene and its aza-derivatives" was retracted in 2026. Reasons: unreliable results or conclusions; concerns about the citations.

#### 3.1.6 Electrophilicity (*ω*) and nucleophilicity (*N*) indices

The electrophilicity index defines the tendency of an electrophile to acquire a given amount of electron density, and the resistance for a molecule to exchange electron density with the surrounding [34]. *ω* is related to *μ* and *Ƞ* as expressed in Eq. (7).

(7) $$\omega =\frac{\mu 2}{2\eta }$$

Organic molecules are classified as strong, moderate and marginal electrophiles depending on the value of electrophilicity index. Strong electrophiles having electrophilicity index >1.5eV, moderate electrophiles have a range of 0.8 < electrophilicity index <1.5eV, while marginal electrophiles are <0.8 eV [41]. The electropositivity index of all the species are closely distributed, except naphthalene, 1-AN and 1,3-DAN. Naphthalene, 1-AN and 1,3-DAN are all marginal electrophile (0.632 eV, 0.632 eV and 0.791 eV respectively), the others are moderate, with 1,4- DAN having the highest electrophilicity index of 0.9766 eV. Organic molecules are classified as strong, moderate and marginal nucleophiles. Molecules with nucleophilicity index: N > 3.0 eV are strong nucleophiles, 2.0 ≤ N ≤ 3.0 eV are moderate, while those with N < 2.0eV are marginal nucleophiles [34]. From Table 2 Naphthalene, 1-AN and 1,2-DAN are strong nucleophiles (N = 3.0041, 3.0041 and 3.2501 eV respectively). The rest compounds are moderate nucleophiles, with 1,6-DAN having the least N value of 2.3794 eV.

### 3.2 Local reactivity descriptors

#### 3.2.1 Condensed fukui function (f) and dual descriptor, (CDD)

The Fukui function values indicate the most probable sites for electrophilic (f^−^) or nucleophilic (f^+^) attacks about a molecule [34]. Calculations for f^−^, f^+^ and f^+^ were carried out using Multiwfn software [27]. For the different atoms present in the various species. From Table S1 of the supporting information. C1, C6 and C9 of naphthalene gave the highest value (0.0899) of f^−^ for naphthalene atoms, indicating that they are the most susceptible to electrophilic attack. On the other hand, C1, C6, C7, and C10 gave f^+^ value of 0.0841 (highest in the group), hence are prone to nucleophilic attack. The f^−^ values for all nitrogen sites in 1-AN, 1, 2-DAN, 1, 3-DAN, 1, 4-DAN, 1, 5-DAN, 1, 6-DAN, 1, 7-DAN and 1, 8-DAN are relatively the least in their corresponding groups, showing that they are almost passive to electrophilic reagents. This could be further explained by the absence of proton on the nitrogen atoms, which makes the good Lewis bases. Alternatively, the f^+^ values for nitrogen sites are highest in the various groups, which explains their high reactivity with electrophiles. The availability of lone pair of electrons, coupled with their conjugated systems improve the electron density around nitrogen, hence a good chemistry with electrophilic reagents. 1-AN, 1, 2-DAN and 1, 3-DAN nitrogen sites gave the highest f^+^ values (1-AN; f^+^ = 0.1012, 1, 2-DAN; f^+^ = 0.1106 for N9 and 0.1102 for N10, while 1, 3-DAN; f^+^ = 0.1294 for N9 and 0.1265 for N10). 1-AN, 1, 2-DAN and 1, 3-DAN are highly susceptible to electrophilic attack when compared to their counterparts, with 1, 3-DAN standing out.

The article "Aromaticity indices, electronic structural properties, and fuzzy atomic space investigations of naphthalene and its aza-derivatives" was retracted in 2026. Reasons: unreliable results or conclusions; concerns about the citations.

The Dual Descriptor is a parameter used in defining the nature of a local site in a molecule as electrophilic (when positive) or nucleophilic (when negative). The CDD values of all species were calculated. Naphthalene gave a positive CDD values at C9 and C10, indicating that naphthalene is electrophilic at these sites. Negative values of CDD were ascertained for all nitrogen sites, showing their nucleophilic properties. Due to high electron density around unsaturated nitrogen sites, which are confirmed by the CDD values from VEDA calculations, they tend to show strong affinity for electron deficient moieties. The highest nucleophilic nitrogen sites are those of 1,6-DAN and 1,7-DAN (CDD for N10 = -0.0912 in 1, 6-DAN and N10 = 0.0941 IN 1, 7-DAN) as can be seen in Table SB of the supporting information.

#### 3.2.2 Local electrophilicity, ω_k_ and nucleophilicity, N_k_

Local electrophilicity and nucleophilicity indices are good parameters in the prediction of regio- and chemo-selectivity in polar chemical interactions [34, 35, 36]. This is achievable because they predict the most electrophilic and nucleophilic centers in molecules. All nitrogen sites exhibited the highest values of nucleophilicity indices in their corresponding molecules, showing an agreement with the dual descriptor values.

The article "Aromaticity indices, electronic structural properties, and fuzzy atomic space investigations of naphthalene and its aza-derivatives" was retracted in 2026. Reasons: unreliable results or conclusions; concerns about the citations.

#### 3.2.3 Condensed local softness

From the local softness values in Table S2, it could be noticed that the nitrogen sites are the softest in each molecule except in 1,4-DAN. Higher values of S^−^ indicates a higher susceptibility to chemical reaction. C1, C6 and C7 with S^−^ values of 0.2661, as can be seen in Table S2 of the supporting information, are the softest sites in normal naphthalene molecule.

### 3.3 Aromaticity indices

Aromaticity of organic compounds is one of the most important characteristics related to their specific chemical reactivity structure [37]. The definition of aromaticity is enumerative in nature [38]. This is because it is described by a collection of physicochemical properties determining specific features of cyclic or polycyclic π-electron molecules [38].

In this study, we used seven indicators which geometry based of aromaticity. The main aim of these descriptors is to measure the amount of electron delocalization, which is associated with the aromaticity of the ring. First, the para-delocalization index (PDI) is calculated as an average of all delocalization index of para-related atoms. The aromatic fluctuation index (FLU) takes into account, the amount of electron sharing between bonded pairs of atoms and the similarity between adjacent atoms, FLU-π which is based on DI-π and π-atomic valence, the para-linear response (PLR) reflects the impact of para perturbation of external potential on the electron density [27]. Table 4 presents the values obtained using the Multiwfn [27] of the studied compounds. Obviously the larger the PDI, the larger the delocalization and the stronger the aromaticity, whereas the lower the FLU, FLU-π and PLR, the stronger the aromaticity [30]. The diazanaphthalenes showed larger PDI, but lower FLU, FLU-π and PLR values and hence more aromatic [30]. Specifically, 1,2-DAN, 1,4-DAN and 1,8-DAN showed more correlations.

To further determine the reliability of the trend shown by the shown by the indices, harmonic oscillator measure of aromaticity (HOMA), BIRD index, and the localized orbital location integrated pi over plane (LOLIPOP), which are geometry-based parameters used to determine the extent at which at which the discussed indices were able to describe the geometry-based aromaticity of the studied compounds. This is one of the best methods to describe the change in aromaticity [23]. If HOMA is unity [22], it means the compound is fully aromatic, while if HOMA equals zero (0), the compound or ring is completely non-aromatic.

The article "Aromaticity indices, electronic structural properties, and fuzzy atomic space investigations of naphthalene and its aza-derivatives" was retracted in 2026. Reasons: unreliable results or conclusions; concerns about the citations.

Inspection of Table 4, reveals that 1,2-DAN, 1,3-DAN, 1,7-DAN and 1,8-DAN exhibited HOMA = 1.0, thus they are geometrically iso-aromatic to each other. Although, the general correlation of the aromaticity parameters investigated seems to be regular, the aromaticity of the diazanaphthalenes are higher. The substitution of the carbon atoms in the ring system and aromaticity changes are connected with the π-electron delocalization. The aromaticity of naphthalene is significantly influenced by the substitution of the carbon atoms with nitrogen.

The indices in Table 3, shows that the diazanaphthalene isomers are more aromatic than naphthalene [37], with 1,7-DAN showing more aromaticity. This is evident as both the Flu, Flu-π, PLR values of about unity (1). Compounds having aromatic indices of 1 are strongly aromatic [38, 39]. Relative aromaticity trend among the analyzed compounds is thus; 1,7-DAN > 1, 8-DAN > 1, 5-DAN > 1, 6- DAN >1, 4-DAN > 1, 2-DAN > 1-AN > naphthalene. Further investigations were carried out to determine the quantitative aromaticity indices of the studied compounds by the determining the harmonic oscillator measure of aromaticity (HOMA), (BIRD) and the non-covalent interaction between aromatic rings using the local orbital locator integrated pi over plane (π-π) (LOLIPOP). The results are presented in Table 4.

**Table 3:** Aromaticity indices values for the various C and N atoms in Naphthalene, 1-AN, 1, 2-DAN, 1, 3-DAN, 1, 4-DAN, 1, 5-DAN, 1, 6-DAN, 1, 7-DAN and 1, 8-DAN.

S/N	Compounds	PDI	FLU	FLU-π	PLR
1	Naphthalene	0.163	0.127	0.621	0.487
2	1-AN	0.887	0.094	0.513	0.789
3	1,2-DAN	1.000	0.734	0.137	0.784
4	1,3-DAN	0.492	0812	0.118	0.521
5	1,4- DAN	1.892	0.596	0.079	0.473
6	1,5- DAN	1.058	0.785	1.133	0.452
7	1,6- DAN	0.694	0.793	0.909	0.779
8	1,7- DAN	0.121	1.401	1.404	0.872
9	1,8- DAN	1.080	0.873	0.457	0.833

The HOMA values of 1 as shown in Table 4, means strong aromaticity of the Diazanaphthalenes, with 1,7-DAN being more aromatic. This value correlates with the stacking ability of the compounds as indicated by LOLIPOP showing that 1,7- DAN has stronger π-stacking ability, hence more aromatic and most stable.

**Table 4:** HOMA, BIRD and LOLIPOP values for the various C and N atoms in Naphthalene, 1-AN, 1,2-DAN, 1,3-DAN, 1,4-DAN, 1,5-DAN, 1,6-DAN, 1,7-DAN AND 1,8-DAN.

S/N	Compound	HOMA	BIRD	LOLIPOP
1	Naphthalene	0.804	0.963	0.971
2	1-AN	0.513	1.577	1.228
3	1,2-DAN	1.195	1.178	1.113
4	1,3-DAN	1.500	1.610	0.082
5	1,4- DAN	0.570	1.600	0.124
6	1,5- DAN	0.680	0.350	0.343
7	1,6- DAN	0.386	1.263	0.798
8	1,7- DAN	1.500	1.560	1.061
9	1,8- DAN	1.250	0.369	0.493

The article "Aromaticity indices, electronic structural properties, and fuzzy atomic space investigations of naphthalene and its aza-derivatives" was retracted in 2026. Reasons: unreliable results or conclusions; concerns about the citations.

### 3.4 Laplacian bond order analysis

The LBO of C–C, C=C, C–H, C–N bonds in the systems presented in Table 5, predicts the sequential strength of the bonds in the order of C=C > C–C > C–N > C–H. This indicates a good correlation with the bonds, that is LBO exhibits bond strength fairly well. This reveals the polarizability of the bonds [40], in the order of C–H > C–N > C–C > C=C.

**Table 5:** Laplacian bond order results for naphthalene, 1-AN, 1,2-DAN, 1,3-DAN, 1,4-DAN, 1,5-DAN, 1,6-DAN, 1,7-DAN AND 1,8-DAN.

Compound	Bond Order			
	C–C	C=C	C–H	C–N
Naphthalene	1.538	1.538	0.832	-
1-AN	1.542	1.556	0.847	1.306
1,2-DAN	1.546	1.558	0.829	1.339
1,3-DAN	1.531	1.546	0.829	1.339
1,4-DAN	1.542	1.556	0.844	1.330
1,5-DAN	1.541	1.554	0.847	1.554
1,6-DAN	1.551	1.565	0.829	1.312
1,7-DAN	1.561	1.559	0.829	1.312
1,8-DAN	1.552	1.556	0.829	1.116

### 3.5 Electrostatic potential (ESP)

ESP diagrams are used to display the difference in electron density distribution around the compounds under study [41]. The blue colour represents area where the excited state density is larger than the ground state density, while the red region is the reverse. As can be visualized from the ESP diagrams in Figure 3. Electron density is evenly distributed around the naphthalene ring without any noticeable distortion. For the analyzed nitrogen derivatives, intense blue colouration surrounds the N sites, showing that electron density moves from other parts of respective compound towards the nitrogen moiety during a transition from the ground state to the first excited state.

**Figure 3:** ESP diagrams for naphthalene, 1-AN, 1,2-DAN, 1,3-DAN, 1,4-DAN, 1,5-DAN, 1,6-DAN, 1,7-DAN AND 1,8-DAN.

### 3.6 OPDOS and PDOS analysis

Density of state (DOS) graph can be used as an important tool for analyzing the nature of electronic orbital mixing for bonding. The vertical dashed line that runs from top to bottom on the graph indicates the position of the HOMO of the molecule under investigation. Also, the polarity of the overlap partial density of states (OPDOS) at any point of the graph defines the bonding behaviour of the orbitals at that point. A negative OPDOS values represents an anti-bonding character for the molecular orbitals (MOs), while a positive value indicates bonding character [42]. While plotting the DOS for the different species, fragment 1, 2 and was defined to represent nitrogen moieties, the carbon atoms, and the hydrogen environment respectively. From the DOS plots reported in Figure 4, it can be visualized for naphthalene that Frag. 1 and 2 have totally different contributions to the electronic system. Frag. 1 exhibited positive values unlike frag. 2. Which dived into the negative side on few occasions. OPDOS at HOMO for naphthalene is at zero. OPDOS for 1-AN, 1,2-DAN, 1,3-DAN, 1,4-DAN, 1,5-DAN, 1,6-DAN, 1,7-DAN and 1,8-DAN evidently gave negative values at their respective HOMO positions, showing anti-bonding properties for MOs at that point. Frag. 1 and 3 gave a comparable amount of contribution for all nitrogen molecules, as shown by the similarities in their pattern.

The article "Aromaticity indices, electronic structural properties, and fuzzy atomic space investigations of naphthalene and its aza-derivatives" was retracted in 2026. Reasons: unreliable results or conclusions; concerns about the citations.

**Figure 4:** PDOS plots for naphthalene, 1-AN, 1,2-DAN, 1,3-DAN, 1,4-DAN, 1,5-DAN, 1,6-DAN, 1,7-DAN AND 1,8-DAN.

### 3.7 Scanning tunnelling microscopy (STM)

Here the STM simulation which was used to study the surface atomic structural pattern of the compounds were simulated using the Multiwfn software as reported in Figure 5. The simulation was performed at voltage bias and current of -0.5 V and 1.2 A respectively.

**Figure 5:** STM diagrams for naphthalene, 1-AN, 1,2-DAN, 1,3-DAN, 1,4-DAN, 1,5-DAN, 1,6-DAN, 1,7-DAN AND 1,8-DAN.

### 3.8 Natural bond orbital (NBO) analysis

In other to depict information about nature of hydrogen bonding and their interactions among bonds, conjugate interactions of molecular systems, NBO analysis was carried out using Gaussian 09 [24] and results analyzed using UCA Fukui [26]. Table S3, shows the natural orbital occupancies and hybrid of the election donor orbitals. The occupancy of an orbital indicates its electrons density. The result from the analyzed compounds indicates that the orbital with the highest occupancy is found in 1,6-DAN σC_6_-N_9_ with occupancy 1.98694 for a hybrid sp^2.05^ and contributed by s(38.24%) p(67.11%), d(0.10%) atomic orbitals and the orbital with the lowest occupancy is found in 1,2-DAN σ∗C_1_–C_2_ with occupancy of 0.21916 for a hybrid sp^1.00^ and contributed by s(0.00) p(99.94) d(0.06) atomic orbitals. The high occupancy found in the 1,6-DAN bonding σC_1_-C_2_ orbital and the low occupancy value found in the anti-bonding σ∗C_1_–C_2_ orbital of 1,6-DAN. This agrees with the findings of Eric D. et al which asserts that bonding (BD) orbitals have high transition energies and anti-bonding orbitals (BD) have low transition energies. The trend in the electron occupancy values across the analyzed compounds show that carbon to N9 (C_X_-N_9_) σ bonds have the highest occupancy values while carbon 1 to carbon 2 (C1–C2) anti-bonding π orbitals have the lowest occupancy values. The high occupancy values found between C–N9 bonds can be attributed to the delocalization of the lone pair electrons of the N9 atom in the molecules and the strong sigma(σ) bond which exist between N9 and the carbon atoms.

Table S4, depicts the second order perturbation theory analysis results of analyzed compounds using B3lyp/6-311+G functional. It shows the various possible donors and acceptors in the most interactive bonds of the naphthalene nitrogen derivatives with their occupancy values in each position as well as their various possible interaction energies between the donor and acceptor orbitals. The stabilization energy for these interactions indicates the highly probable and low probable interactions in the molecules. The analyzed results reveal that the 3 highest transition energies in the molecules are C_6_–N_a_ to C_3_–C_4_ $(\pi^{*}-\pi^{*}$ 236.90 kcal/mol) of 1,6-DAN, C_3_–C_4_ to C_1_–C_2_ ($\pi^{*}-\pi^{*}$236.37 kcal/mol) of 1-AN and C_7_–N_10_ to C_2_–C_4_ ($\pi^{*}-\pi^{*}$235 kcal/mol) of 1,3-DAN. The lowest stabilization energies in the molecules are found in 1,4-DAN; C_8_–N_10_ to C_7_–C_8_ (σ -σ∗ 1.26 kcal/mol), 1,5-DAN; C_3_–C_9_ to C_5_–C_8_ (σ - σ ∗2.04 kcal/mol) and 1, 2-DAN; C3–N9 to C3–C5 (2.05 Kcal/mol). These result reveals that the highest stabilization energies exist between the $\pi^{*}\;to\;\pi^{*}$(pi anti bonding) orbitals and this is due to the strong π bonds and the anti-bonding orbitals which increases the energy of the molecule. These high interaction energies give stability to the compound.

The article "Aromaticity indices, electronic structural properties, and fuzzy atomic space investigations of naphthalene and its aza-derivatives" was retracted in 2026. Reasons: unreliable results or conclusions; concerns about the citations.

## 4 Conclusion

In this study, the aromaticity, electronic structural properties of naphthalene and its aza-derivatives were computationally studied. The results obtained convincingly showed that the azanaphthalenes are more aromatic and more stable as described by the electronic structural properties. Observed trend is in line with the fact that an increase in electron density renders a molecule π-deficient, hence the diazanaphthalene are prone to nucleophilic attack. This observed trend could be used to study biological activities of the most stable isomers of the diazanaphthalenes.

## Declarations

### Author contribution statement

Moses Mbeh Edim: Conceived and designed the experiments; Analyzed and interpreted the data; Wrote the paper.

Hitler Louis: Conceived and designed the experiments.

Obieze C. Enud, Bassey B. Asuquo, Emmanuel A. Bisong, John A. Agwupuye, Gloria C. Apebende, Innocent Joseph, Joseph O. Odey: Performed the experiments; Analyzed and interpreted the data.

Francisca I. Bassey: Contributed reagents, materials, analysis tools or data.

### Funding statement

This research did not receive any specific grant from funding agencies in the public, commercial, or not-for-profit sectors.

### Data availability statement

The authors do not have permission to share data.

### Declaration of interests statement

The authors declare no conflict of interest.

### Additional information

No additional information is available for this paper.

The article "Aromaticity indices, electronic structural properties, and fuzzy atomic space investigations of naphthalene and its aza-derivatives" was retracted in 2026. Reasons: unreliable results or conclusions; concerns about the citations.

## Appendix A Supplementary data

Supporting_information_moses_spl_1_spl_ Supporting_information_moses_spl_1_spl_
